# Mechanisms of Kidney Cell Pyroptosis in Chronic Kidney Disease and the Effects of Traditional Chinese Medicine

**DOI:** 10.1155/2021/1173324

**Published:** 2021-10-11

**Authors:** Baozhu Ding, Guoping Ma, Zinuo Wang, Wenjie Liang, Weifang Gao

**Affiliations:** ^1^College of Integrated Traditional Chinese and Western Medicine, Hebei University of Chinese Medicine, Shijiazhuang, Hebei, China; ^2^Hebei Key Laboratory of Integrative Medicine of Liver-Kidney Patterns, Institute of Integrative Medicine, Hebei University of Chinese Medicine, Shijiazhuang, Hebei, China; ^3^The First Hospital, Hebei Medical University, Shijiazhuang, Hebei, China; ^4^College of Pharmacy, Hebei University of Chinese Medicine, Shijiazhuang, Hebei, China

## Abstract

Chronic kidney disease (CKD) is a major public health issue that is highly prevalent worldwide. Pyroptosis is an important pathological mechanism underlying kidney cell damage in CKD and is associated with the classic caspase-1-mediated pathway and nonclassic caspase-4/5/11-mediated pathway. The NLRP3-caspase-1-GSDMD signaling pathway is the key mechanism of kidney cell pyroptosis in CKD, and noncoding RNAs such as lncRNAs and miRNAs are important regulators of kidney cell pyroptosis in CKD. In addition, the NLRP1/AIM2-caspase-1-GSDMD and caspase-3-GSDME signaling pathways have also been shown to mediate kidney cell pyroptosis. Traditional Chinese medicine (TCM) and extracts can interfere with the occurrence and development of kidney cell pyroptosis in CKD by inhibiting the NLRP3 signaling pathway and oxidative stress, activating Nrf-2 signaling, protecting mitochondrial integrity, regulating AMPK signaling, and regulating TXNIP/NLRP3 axis, which have become increasingly prominent. It is critical to explore the effects of TCM on kidney cell pyroptosis in CKD and its mechanisms to identify targets and develop new and effective drugs.

## 1. Introduction

Chronic kidney disease (CKD) is recognized as a major public health concern. According to a report published in *The Lancet* in 2020, CKD is still a highly prevalent disease worldwide, affecting 9.1% of the world's population. In 2040, this number is estimated to increase to 2.2–4 million. The number of CKD patients in China has reached 132.3 million, the incidence is as high as 10.8% [1], and many CKD patients are more likely to progress to end-stage renal disease, seriously endangering public health [2]. Thus, early detection and intervention are crucial for CKD patients. However, no specific drug is available to reverse or block the progression of CKD, and the pathogenesis remains largely elusive. Several studies [3] have shown that CKD is closely related to inflammation. Cellular pyroptosis is an important mechanism associated with inflammatory damage to renal tissue and progression in CKD, which is an inflammatory disease.

Pyroptosis, also known as inflammatory apoptosis, is a mode of programmed cell death that relies on cysteine-containing aspartate-specific proteases (Caspases). Pyroptosis possesses some characteristics of apoptosis and necrosis, including the basic characteristics of DNA damage and membrane damage [4]. During pyroptosis, several kinds of pathogen-associated molecular patterns (PAMPs) and damage-associated molecular patterns (DAMPs) trigger inflammasome formation, which activates caspases, thereby cleaving gasdermin D (GSDMD) or gasdermin E (GSDME), the effector proteins of pyroptosis. These cleaved gasdermins bind with the lipids of the cell membrane to form membrane pores and cause pyroptosis [5].

Pyroptosis is widely involved in the occurrence and development of kidney, infectious, and atherosclerotic diseases [6–8]. CKD is a serious threat to human health. Currently, no effective medicine or desirable method is available to reverse or block the progression of CKD; therefore, it is urgent to find novel treatment approaches and drugs [9]. Through syndrome differentiation and treatment, traditional Chinese medicine (TCM) has exhibited good efficacy in the treatment of CKD, and the effects of TCM on pyroptosis have become increasingly prominent [10]. Exploring the effects and mechanisms of TCM on CKD-associated pyroptosis is of great importance in pathological research, clinical prevention, and the development of new drugs.

## 2. Pyroptosis and CKD

Pyroptosis can occur and develop in various CKDs, such as diabetic nephropathy (DN), obstructive nephropathy, renal fibrosis, and crystal-related nephropathy. The mechanisms underlying pyroptosis include classic and nonclassic pathways [11, 12].

### 2.1. The Classic Pyroptosis Pathway in CKD

Caspase-1-dependent cell death is known as a classic pyroptosis pathway [11, 13]. The caspase family is typically divided into two subfamilies, apoptotic caspases and inflammatory caspases, which play important roles in innate immunity and include caspase-1, 4, 5, 11, and 12 [14]. Caspase-1 is the main mediator of pyroptosis. The inflammasomes involved in the classic pyroptosis pathway in CKD mainly include NOD-like receptor protein 3 (NLRP3) and NLRP1 and absent in melanoma 2 (AIM2) inflammasomes [13].

#### 2.1.1. The NLRP3 Inflammasome Signaling Pathway

The inflammasome, also known as the pyroptotic body [15], is a complex formed by the assembly of multiple proteins, such as pattern recognition receptor (PRRs), in cells. Inflammasomes are generally composed of receptor molecules, adapter molecules, and effector molecules. Receptor molecules include NOD-like receptor (NLR) family molecules and AIM2-like receptor (ALR) family molecules. The former are the most important type of PRR [16] and include 14 members of the NLRP subfamily (NLRP1–NLRP14) and NLRC4 [17].

The receptor molecule of the NLRP3 inflammasome is NLRP3. The adapter molecule is called apoptosis-related punctate protein with caspase activation and recruitment domains (ASC), and the effector molecule is caspase-1 [18]. PAMPs are expressed by CKD-associated pathogens, and DAMPs are released by chronic renal damage and include extracellular matrix components such as reactive oxygen species (ROS), extracellular ATP, uric acid, and disaccharides [17, 19]. PAMPs and DAMPs activate NLRP3, which oligomerizes to form the NLRP3 complex; the complex then recruits procaspase-1 monomers through the adapter protein ASC, activating caspase-1. Caspase-1 processes the proinflammatory cytokine pro-IL-1*β*/pro-IL-18 to generate mature IL-1*β*/IL-18, which is released by cell lysis during pyroptosis [20]. GSDMD is cleaved to produce N-terminal GSDMD (GSDMD-NT), which binds to lipids in cell membranes to form pores of 1 to 2 nm and initiate pyroptosis. Pyroptosis is characterized by cell swelling and high permeability of the plasma membrane followed by lysis and the release of cytoplasmic contents, which trigger necrotizing inflammation [3]. Pyroptosis promotes the extracellular release of IL-1*β*/IL-18, initiates the inflammatory response, and promotes the release of intracellular DAMPs, further inducing pyroptosis in other cells and forming a positive feedback loop, thereby exacerbating inflammation-mediated kidney damage [21]. The specific mechanism is shown in (1) in Figure 1. Pyroptosis is mediated by the NLRP3/caspase-1/GSDMD signaling pathway and is an important mechanism of inflammatory renal injury in CKD [18, 21]. In renal macrophages, podocytes, endothelial cells, and other intrinsic cells, the NLRP3 inflammasome can be activated to promote inflammatory responses and accelerate the progression of CKD [22]. Studies [18, 23] have shown activation of the NLRP3 inflammasome in various CKDs, such as obstructive nephropathy, chronic type II crystalline nephropathy, DNP, lupus nephritis, and IgA nephropathy, further exacerbating kidney damage. However, no NLRP3 antagonists have been approved for treatment to date, and there is an urgent need for specific NLRP3 inhibitors, which would provide a wide range of therapeutic potential for the treatment of CKD.

#### 2.1.2. The NLRP1 Inflammasome Signaling Pathway

The NLRP1 inflammasome is composed of NLRP1, ASC, and caspase-1 [24]. As ligands of NLRP1, bacterial muramyl dipeptide, anthrax toxin, toxoplasma gondii, etc., can activate the NLRP1 inflammasome [25]. The specific mechanism is shown in (2) in Figure 1. Yu et al. [4] reported that high glucose and high insulin induced NLRP1 inflammasome activation in glomerular mesangial cells and that caspase-1 expression was upregulated, which led to pyroptosis and an inflammatory response. Downregulating NLRP1 could inhibit pyroptosis. NLRP1 contains a C-terminal CARD, which can be directly activated by interacting with the CARD of procaspase-1 [20], but ASC transduction can enhance the activity of procaspase-1. However, Finger et al. reported that NLRP1 was activated in an ASC-dependent manner [19, 26].

#### 2.1.3. The AIM2 Inflammasome Signaling Pathway

The AIM2 inflammasome is composed of AIM2, ASC, and caspase-1 [27]. The dsDNA released by pathogens or kidney damage is an AIM2 ligand. dsDNA can bind to and activate the C-terminal HIN200 domain of AIM2 [28], and the PYD domain of activated AIM2 molecule interacts with that of ASC molecule to activate ASC. The activated CARD of ASC binds with the CARD of procaspase-1 to assemble and form the AIM2 inflammasome [20], and procaspase-1 cleaves and activates itself, eventually causing pyroptosis [20, 29]. The specific mechanism is shown in (3) in Figure 1. Sharma et al. [30] showed that acute kidney injury leads to tubular cell necrosis and the release of DNA, which is taken up by neighboring macrophages. The AIM2 inflammasome is then activated, leading to the production of proinflammatory cytokines, such as IL-1*β* and IL-18, thereby promoting chronic kidney inflammation. Komada et al. [31] found that in the course of CKD, DNA from damaged cells was the main DAMP, activating the AIM2 inflammasome in macrophages and leading to pyroptosis and the promotion of inflammation to accelerate fibrosis. Other DAMPs can simultaneously activate the NLRP3 inflammasome, exacerbating the occurrence of pyroptosis.

### 2.2. The Nonclassic Pyroptosis Pathway in CKD

The mode of cell death that relies on caspase-4/5/11 is the nonclassic pyroptosis pathway [12]. Human caspase-4/5 and mouse caspase-11 serve the same function. When a pathogen invades kidney cells, lipopolysaccharide (LPS), also known as lipid A, binds to and activates the CARD of caspase-11 [32], which then cleaves GSDMD and induces pyroptosis. Moreover, the gap junction protein 1 (pannexin 1) transmembrane channel is cleaved, forming a pathway through which intracellular ATP is released. ATP binds to the membrane receptor P2X7, opening the nonselective P2X7 positive ion channel, which causes intracellular K+ efflux, extracellular Na+ and Ca2+ influx, and ultimately cell membrane damage, leading to pyroptosis [33–35]. The specific mechanism is shown in (4) in Figure 1. Yang et al. [36] found that ischemia-reperfusion could induce caspase-11-mediated pyroptosis in renal tubular epithelial cells in mice. The caspase-11-mediated nonclassic pyroptosis pathway leads to intracellular DAMP release and K^+^ efflux, which activates the NLRP3 inflammasome and induces the classic, caspase-1-mediated pyroptosis pathway. Furthermore, inflammatory cytokines such as IL-1 are released to exacerbate inflammatory injury. Caspase-11 gene knockout can reduce the expression of LPS-induced pyroptosis-related proteins and the release of inflammatory factors in renal tubular epithelial cells, thereby reducing the progression of CKD [37, 38].

In addition, it was recently discovered that the caspase-3/GSDME signaling pathway could also induce pyroptosis. GSDME is another gasdermin family protein [28]. Zeng et al. [39] found that when the classic NLRP3 signaling pathway was blocked, ATP could activate caspase-3 in macrophages and lyse GSDME, leading to GSDME-NT production, membrane pore formation, and the resulting pyroptosis. The specific mechanism is shown in (5) in Figure 1. Through animal experiments and cell culture, Li [40] demonstrated that caspase-3 could specifically cleave GSDME to induce kidney cell pyroptosis in DN. Zhou's [41] Western Blot test confirmed that BSA can induce the exposure of GSDME-NT, a protein related to early cell pyroptosis. The activation of NLRP3 inflammasome may mediate the pyroptosis of kidney NRK-52E cells induced by BSA. Caspase-3 cuts GSDME and exposes GSDME-NT, thereby inducing cell death by pyroptosis before apoptosis. Tu [42] found that Huaier, a traditional Chinese medicine, can regulate the pyroptosis of mesangial cells by inhibiting the caspase-3/GSEME signaling pathway, reducing the release of inflammatory factors, and exerting renal protection. Wang [43] showed that TNF-*α* and chemotherapy drugs could activate the caspase-3/GSDME pathway in cancer cells and induce pyroptosis. Thus, the role of caspase-3-GSDME in CKD pyroptosis is important for future research.

### 2.3. The Regulatory Mechanism of Noncoding RNAs in Kidney Cell Pyroptosis in CKD

Long noncoding RNAs (lncRNAs) and microRNAs (miRNAs), as well as other noncoding RNAs, are important regulators of kidney cell pyroptosis in CKD [44]. As novel nonprotein gene expression regulators, miRNAs play important roles in CKD, and lncRNAs can improve CKD by regulating miRNA expression [45].

#### 2.3.1. MALAT1 and miR-23c/miR-30c

Metastatic-associated lung adenocarcinoma transcript 1 (MALAT1) and miR-23c/miR-30c belong to the lncRNA and miRNA families, respectively. It was found that in the pathogenesis of diabetic nephrosis (DN), MALAT1 and miR-23c are characterized by pro- and antipyroptotic properties, respectively [46]. MALAT1 can trap miR-23c and downregulate the expression of miR-23c, while the target gene of miR-23c is the pyroptosis-related protein ELAV-like protein 1 (ELAVL1). The upregulation of ELAVL1 can induce the expression of NLRP3 and other downstream pyroptosis-related molecules, resulting in pyroptosis. MALAT1 expression was significantly increased in the kidneys of STZ-induced diabetic rats and HK-2 cells treated with high glucose, whereas the expression of miR-23c was significantly decreased, leading to the upregulation of ELAVL1 and downstream pyroptosis-related molecules. Therefore, the expression of ELAVL1, NLRP3, caspase-1, and IL-1*β* in DN kidneys was positively regulated by MALAT1 and negatively regulated by miR-23c. Liu et al. [47] found that MALAT1 can also inhibit miR-30c targeting NLRP3 through a similar pathway to regulate the pyroptosis of renal tubular epithelial cells induced by high glucose.

#### 2.3.2. GAS5 and miR-452-5p

Growth arrest-specific transcript 5 (GAS5) and miR-452-5p belong to the lncRNA and miRNA families, respectively. Unlike MALAT1 and miR-23c, GAS5 possesses antipyroptotic properties, while miR-452-5p, the target molecule of GAS5, has propyroptotic properties.

In human tubular epithelial cells (HK-2) induced by high glucose, the classic pyroptosis signaling pathway is activated. Therefore, ROS, NLRP3, caspase-1, IL-1*β*, GSDMD-NT, and other pyroptosis-related molecules, as well as IL-6, TNF-*α*, MCP-1, and other inflammatory factors and miR-452-5p, are significantly upregulated, and GAS5 is downregulated. MiR-452-5p interference can inhibit the expression of pyroptosis-related molecules. GAS5 directly targets miR-452-5p, and high GAS5 expression can inhibit high glucose-induced pyroptosis in renal tubular epithelial cells by downregulating the expression of miR-452-5p [45].

Table 1 summarizes the different types of pyroptosis in kidney cells.

## 3. Effects of Traditional Chinese Medicine or Extracts

### 3.1. Regulation of the NLRP3/Caspase-1/IL-1*β* Signaling Pathway

The main mechanism of pyroptosis in CKD is the classic pathway, which is mediated by the NLRP3 inflammasome. TCM or extracts can directly or indirectly inhibit NLRP3 signaling pathway molecules and pyroptosis, slowing the development of CKDs, such as DN, obstructive nephropathy, and lupus nephropathy. Liang et al. [10] reported that huayu jiedu recipe (HJR) (*Astragalus membranaceus*, vinegar turtle shell, batryticated silkworm, black tip snake, earthworm, radix paeoniae rubra, *Salvia miltiorrhiza*, radix scutellariae, honeysuckle, dandelion, and rhubarb) could downregulate mDCT-induced NLRP3 inflammasome expression in rat kidneys with unilateral ureteral obstruction (UUO) and renal tubular epithelial cells, regulate the NLRP3-caspase-1-IL-1*β*axis/IL-18 axis, inhibit pyroptosis, and antagonize inflammatory lesions, thus slowing the progression of obstructive nephropathy. Wang et al. [51] discovered supplemented Gegen Qinlian decoction formula (SGDF), composed of *Pueraria lobata*, *Coptis*, *Scutellaria*, raw licorice, rhubarb, and cinnamon. It can improve the degree of immunostaining of NLRP3, caspase-1, GSDMD-N, and IL-1*β* in the glomerulus of diabetic nephropathy model mice and the protein expression level in kidney tissue, thereby reducing podocyte pyroptosis. Guo Xiaoyuan [52] found that Zi Shen Wan (ZSW: composed of *Phellodendron amurense*, Anemarrhena, and cinnamon) can reduce the pyroptosis of renal tubular epithelial cells in db/db mice by inhibiting the activation of NLRP3 inflammasomes and can effectively inhibit the mesenchymal changes, and the migration ability of HK-2 cells induced by high glucose can reduce nuclear damage and cell membrane damage, inhibit the expression of pyroptosis-related inflammatory factors, and reduce early renal damage in DN. Feng et al. [53] found that the Yiqi Jianpi Xiezhuo decoction (consisting of *Astragalus*, *Angelica,* white peony root, yam, mulberry parasitic, dogwood, *Smilax*, and *Alisma*) can inhibit the activation of NLRP3 inflammasomes and inhibit renal cell pyroptosis, reduce kidney inflammation damage, and alleviate kidney inflammation damage in pregnant rats with chronic kidney disease. Zhao et al. [54] found that ginsenoside Rh2 is an effective component of traditional Chinese medicine ginseng, which can improve DN kidney damage by regulating caspase-1-mediated cell pyroptosis. Quercetin is the active ingredient of the Chinese herbal medicines *Bupleurum* root, mulberry leaf, locust horn, spiral flower, and hawthorn that has anti-inflammatory, antioxidant, and anticancer effects. Hu et al. [55] found that quercetin could downregulate the expression of renal NLRP3, ASC, and caspase-1, inhibit activation of the NLRP3 inflammasome, and improve the accumulation and damage of renal lipids under increased uric acid conditions and hyperlipidemia.

### 3.2. Inhibition of Oxidative Stress

Oxidative stress is a cellular stress response caused by ROS or the relative overload of free radicals [56]. ROS mainly refer to oxygen-containing compounds whose chemical properties are more active than those of oxygen. Disturbances in the homeostasis of oxidative and antioxidative systems give rise to excessive ROS production, weakened superoxide dismutase (SOD) activity, and increased lipid peroxide (LPO) production. SOD is the main scavenger of oxygen free radicals in the body and can protect cells from oxidative stress damage. SOD activity indirectly reflects the body's ability to remove ROS. LPO is the product of ROS attack of polyunsaturated fatty acids in phospholipids in biofilms and induce lipid peroxidation, which can reflect the degree and rate of lipid peroxidation. Given insufficient antioxidant capacity, ROS can induce oxidative stress and activate the NLRP3 inflammasome, leading to caspase-1-mediated pyroptosis. Chronic inflammation and oxidative stress play key roles in the development of CKD.

Neferine is an effective component of lotus seed embryos and has biological properties such as antioxidant and anti-inflammatory effects. High glucose can induce oxidative stress in mesangial cells in DN [57]. Neferine can inhibit the production of ROS, increase the activity of SOD, and inhibit LPO. Neferine has a free radical scavenger-like effect, and ROS are activators of the NLRP3 inflammasome. By regulating ROS, neferine inhibits oxidative stress and activation of the NLRP3/caspase-1 signaling pathway to inhibit pyroptosis, thereby providing a basis for the treatment of CKD [58]. Trehalose from the TCM seaweed and *Psidium guajava* from plant-based herbal medicines also exert antioxidant effects. The combination of these two treatments can reduce the level of IL-*β*-induced inflammation in the kidney in diabetic rats by reducing the type 2 diabetes-induced ROS levels in kidney tissue, thus inhibiting kidney cell pyroptosis and exerting a protective effect on the kidneys [59].

### 3.3. Activation of Nrf-2 Signaling

Nuclear factor erythroid-2-related factor 2 (Nrf-2), the most important regulator of oxidative stress [60], regulates the expression of protective antioxidant genes to reduce systemic oxidative overload [61], thus reducing oxidative stress and inflammation [62]. Sulforaphane, which is an extract of cruciferous plants such as broccoli, kale, and northern carrot, is a common antioxidant. Studies [63] have shown that sulforaphane is an activator of Nrf-2 that can antagonize ROS, inhibit oxidative stress, and activate the NLRP3 inflammasome. Chung et al. [64] reported that UUO-induced oxidative stress and inflammation and exacerbated pyroptosis, but sulforaphane could reduce pyroptosis caused by inflammasome activation and obstructed kidney damage by activating Nrf-2 signaling, increasing nuclear Nrf-2 translocation, promoting antioxidant gene expression, detoxifying ROS, and inhibiting UUO-induced oxidative stress and NLRP3 inflammasome activation.

### 3.4. Protection of Mitochondrial Integrity

Mitochondrial damage can promote the release of mitochondrial DNA, ROS, and other cytoplasmic components, activating the NLRP3 inflammasome and leading to pyroptosis. The mitochondrial inner membrane is rich in highly unsaturated fatty acids but is vulnerable to ROS attack. Therefore, mitochondria are not only the main site of ROS production in vivo but also extremely sensitive to ROS-mediated oxidative damage [65]. Resveratrol is a polyphenol compound extracted from various Chinese herbal medicines, such as *Polygonum cuspidatum*. Ya [66] reported that resveratrol could inhibit mitochondrial damage in macrophages, reduce mitochondrial DNA transposition to the cytoplasm, and inhibit NLRP3 and NLRP1 inflammasome activation, thereby inhibiting the classic caspase-1-mediated pyroptosis pathway and alleviating renal inflammation-induced damage in mice with progressive IgA nephropathy.

### 3.5. Regulation of AMPK Signaling

AMP-activated protein kinase (AMPK) is a pivotal molecule that regulates energy metabolism and affects a series of cellular metabolic processes. AMPK maintains a balance between ATP consumption and production in eukaryotic cells by sensing the energy state of the cell, which is known as energy homeostasis. It was found that [67] AMPK was significantly activated during ATP-induced pyroptosis. AMPK signaling can regulate the activation of inflammasomes and pyroptosis induced by LPS + ATP, and enhanced AMPK activity can significantly promote pyroptosis. Piperine, the active ingredient of the TCM black pepper, has a number of functions, such as antitumor and antioxidative activities. Studies [68] have shown that piperine can block AMPK signaling, significantly inhibit the expression of key molecules in the NLRP3 inflammasome in the kidneys of lupus nephritis mice, inhibit the caspase-1-mediated classic pyroptosis pathway, and reduce the release of proinflammatory cytokines such as IL-1, blocking renal tubular epithelial cell pyroptosis and thereby inhibiting the progression of lupus nephritis. In addition, the AMPK agonist metformin can bypass the activity of piperine and activate NLRP3 inflammasome-mediated recovery of pyroptosis. The specific mechanisms by which AMPK signaling regulates NLRP3 inflammasome activation and pyroptosis still require further investigation.

### 3.6. Regulation of Thioredoxin-Interacting Protein TXNIP/NLRP3 Axis

Thioredoxin-interacting protein (TXNIP) is an oxidative stress regulator protein involved in cell proliferation, differentiation, and apoptosis. TXNIP inhibits its antioxidant activity by combining with the endogenous antioxidant thioredoxin (TRX) [50]. Both TRX and TXNIP are expressed in the cytoplasm and mitochondria. TXNIP is a protein that connects oxidative stress and activates inflammation. It can activate ROS and also induce the production of ROS. The overproduction of mitochondrial ROS is a key factor in the activation of NLRP3 inflammasome. The inflammasome activator can induce the dissociation of TXNIP from TXNIP/TRX in a ROS-dependent manner. The oxidized TRX is in a free state and is easily combined with the leucine-rich repeat sequence structure of NLRP3, leading to the activation of NLRP3 inflammasome. Chi kun [48] found high uric acid can promote the dissociation of TXNIP/TRX through ROS, which in turn leads to the activation of NLRP3 inflammasomes, causing endothelial cell inflammation and pyroptosis.

Polyphenols are natural antioxidants, which are found in various human dietary components, such as fruits, vegetables, and tea, and play a protective role in many chronic diseases, such as diabetes, cardiovascular diseases, and neurodegenerative diseases. Pomegranate is a widely grown and edible fruit that contains many polyphenols. Punicalagin is the main component of pomegranate polyphenols. Abaiset al. [49] showed that excessive production of mitochondrial ROS (mtROS) leads to the separation of TXNIP from its binding protein Trx, which subsequently binds to NLRP3, leading to the activation of NLRP3 inflammasome. Punicarin can reduce pyroptosis by inhibiting the TXNIP/NLRP3 axis, thereby inhibiting the development of DN. Inhibiting the inflammatory response caused by pyroptosis is an important part of punicalagin to protect the kidneys.

Table 2 summarizes the effects of traditional Chinese medicine or extracts on kidney cells pyroptosis in chronic kidney disease.

## 4. Conclusion

Pyroptosis is an important pathological mechanism underlying kidney cell damage in CKD, including classic pyroptosis mediated by caspase-1 and nonclassic pyroptosis mediated by caspase-4/5/11. The NLRP3-caspase-1-GSDMD signaling pathway is the main mechanism of kidney cell pyroptosis in CKD. Noncoding RNAs such as lncRNAs and miRNAs are key regulators of kidney cell pyroptosis in CKD. Herbal compound formulas, TCM extracts, and effective components can suppress kidney cell pyroptosis by inhibiting the expression of the NLRP3 inflammasome and oxidative stress, activating Nrf-2 signaling, protecting mitochondrial integrity, regulating AMPK signaling, and regulating TXNIP/NLRP3 axis.

To date, although specific drugs are not available for the treatment of kidney cell pyroptosis, TCM has achieved remarkable effects in the treatment of CKD. The role of TCM is characterized by multiple targets and complexity. Therefore, in-depth study on the molecular mechanisms of pyroptosis in the occurrence and progression of kidney disease is warranted to provide more objective evidence for clinical treatment and is critical for identifying targets and developing new and effective drugs.

## Figures and Tables

**Figure 1:** Mechanisms of kidney cell pyroptosis in chronic kidney disease. (1) (NLRP3-caspase-1-GSDMD pathway) PAMPs and DAMPs activate NLRP3 molecules, NLRP3 oligomerizing to form the NLRP3 complex, which recruits procaspase-1 monomers through the adapter protein ASC, activating caspase-1. Caspase-1 processes the pro-IL-1*β*/pro-IL-18 to generate mature IL-1*β*/IL-18, and in the meantime, GSDMD is cleaved to produce GSDMD-NT, which damage the cell membrane eventually leading to pyroptosis. Then, IL-1*β* and IL-18 are released extracellularly, initiating the inflammatory response. Simultaneously, pyroptosis promotes the release of intracellular DAMP, further inducing pyroptosis in other cells and forming a positive feedback loop, aggravating renal inflammation damage. (2) (NLRP1-caspase-1-GSDMD pathway) Bacterial muramyl dipeptide, anthrax toxin, etc., can activate the NLRP1 inflammasome. The NLRP1 molecule C-terminal CARD domain can be directly activated by interacting with the CARD domain of procaspase-1, then activating caspase-1. The next steps are similar to the NLRP3 pathway. (3) (AIM2-caspase-1-GSDMD pathway) dsDNA can bind to and activate the C-terminal HIN200 domain of AIM2, and the PYD domain of the activated AIM2 molecule interacts with that of the ASC molecule to activate ASC. The CARD domain of activated ASC combines with the CARD domain of procaspase-1 to form AIM2 inflammasome, and procaspase-1 cuts and activates itself, eventually causing pyroptosis. (4) (LPS-caspase-4/5/11-GSDMD pathway) When the pathogen invades the kidney cells, the component of LPS, lipid A, binds to and activate the CARD domain of caspase-11, thereby cleaving GSDMD and causing pyroptosis. Meanwhile, the gap junction protein 1 (pannexin 1) transmembrane channel is cleaved, forming a pathway, along which the intracellular ATP is released. ATP binds to the membrane P2X7 receptor, opening the nonselective P2X7 positive ion channel, which causes intracellular K+ outflow and extracellular Na+ and Ca2+ inflow, and finally the cell membrane is damaged, leading to pyroptosis. (5) (ATP-caspase-3-GSDME pathway) ATP can activate caspase-3 in macrophages and lyse GSDME protein to produce GSDME-NT. GSDME-NT is similar to GSDMD-NT, leading to membrane pore formation, eventually resulting in pyroptosis.

**Table 1:** Different types of pyroptosis in kidney cells.

Classification		Description	Kidney cells	Mechanism	Signaling pathways	Reference
The classic pyroptosis pathway in CKD	Activate NLRP3 inflammasome signaling pathway	Cultured primary RTE cells, NLPR3 inflammasome induced renal tubular epithelial cells necrosis.	Renal tubular epithelial cells	NLRP3 inflammasome activation	NLRP3-caapse-1-IL-1*β*/IL-18	[48]
		(1) During hyperhomocysteinemia, podocyte injury and glomerular sclerosis are consequences of NLRP3 inflammasome activation. (2) And high glucose treatment in mice induced NADPH oxidase activity, triggering NLRP3 inflammasome activation in glomerular podocytes and leading to podocyte injury during DN.	Podocyte			[23, 49] [22, 50]
	Activate NLRP1 inflammasome signaling pathway	High glucose and high insulin induced NLRP1 inflammasome activation in glomerular mesangial cells.	Glomerular mesangial cells.	NLRP1 inflammasome activation	NLRP1-caspase-1-IL-1*β*	[4]
	Activate AIM2 inflammasome signaling pathway	Kidney injury leads to tubular cell necrosis and the release of DNA, which is taken up by neighboring macrophages, the AIM2 inflammasome is then activated.	Expressed in glomerular and tubular epithelial cells	AIM2 inflammasome activation	AIM2-caspase-1-IL-1*β*/IL-18	[30, 31]
The nonclassic pyroptosis pathway in CKD	Caspase-4/5/11-mediated pyroptosis	Ischemia-reperfusion could induce caspase-11-mediated pyroptosis in renal tubular epithelial cells in mice. Caspase-11 gene knockout can reduce the expression of LPS-induced pyroptosis-related proteins and the release of inflammatory factors in renal tubular epithelial cells.	Renal tubular epithelial cells	Caspase-11 activation	CHOP/LPS-caspase-11-IL-1*β*	[36–38]
	Caspase-3/GSDME mediated pyroptosis	Caspase-3 could specially cleave GSDME to induce kidney cell pyroptosis in DN.	1. Human tubular epithelial cells (HK-2 cells) 2. Glomerular mesenchymal cells (RGMCs cells) 3. Kidney NRK-52E cells	Caspase-3 cleaved GSDME-induced pyroptosis	Caspase-3-GSEME	[40–42]

**Table 2:** Effects of traditional Chinese medicine or extracts on kidney cells pyroptosis in chronic kidney disease.

Traditional Chinese Medicine or extracts	Description	Mechanism of activation	Regulatory mechanisms	Reference
Huayu jiedu recipe (HJR)	Traditional Chinese medicine compound	Rat kidneys with unilateral ureteral obstruction (UUO) and cultivated renal tubular epithelial cells	Regulation of the NLRP3/caspase-1/IL-1*β* signaling pathway	[10]
Supplemented Gegen Qinlian decoction formula (SGDF)		Diabetic nephropathy model mice, reducing podocyte pyroptosis		[51]
Zi Shen Wan (ZSW)		Renal tubular epithelial cells in db/db mice; HK-2 cells induced by high glucose		[52]
Yiqi Jianpi Xiezhuo decoction		Pregnant rats with chronic kidney disease		[53]
Ginsenoside Rh2	An active ingredient of ginseng	Diabetic nephropathy		[54]
Huaier	*Trametes robiniophila Murr*	Mesangial cells in a rat model of nephritis	Caspase-3/GSDME signaling pathway	[42]
Quercetin	The active ingredient of the Chinese herbal medicines	Accumulation and damage of renal lipids under increased uric acid conditions and hyperlipidemia	Downregulate expression of renal NLRP3, ASC, and caspase-1 and inhibit activation of the NLRP3 inflammasome	[55]
Neferine	An effective component of lotus seed embryos	High glucose induce oxidative stress in mesangial cells in DN	By regulating ROS, inhibits oxidative stress	[57, 58]
Trehalose	TCM seaweed	Type 2 diabetes		[59]
*Psidium guajava*	Plant-based herbal medicines			
Sulforaphane	An extract of cruciferous plants	UUO-induced oxidative stress and inflammation	Activating Nrf-2 signaling, increasing nuclear Nrf-2 translocation	[62–64]
Resveratrol	Polyphenol compound extracted from various Chinese herbal medicines	Renal inflammation-induced damage in mice with progressive IgA nephropathy	Inhibit mitochondrial damage in macrophages, reduce mitochondrial DNA transposition to the cytoplasm, and inhibit NLRP3 and NLRP1 inflammasome activation	[66]
Piperine	The active ingredient of the TCM black pepper	Lupus nephritis mice	Block AMPK signaling, inhibit the caspase-1-mediated classic pyroptosis pathway, and block renal tubular epithelial cell pyroptosis	[68]
Punicalagin	The main component of pomegranate polyphenols	Diabetic nephropathy	Reduce pyroptosis by inhibiting the TXNIP/NLRP3 axis	[49]

## Data Availability

All data used to support the findings of this study are included within the article.
